The article "Disorder-related risk factors for revision total hip arthroplasty after hip hemiarthroplasty in displaced femoral neck fracture patients: a nationwide population-based cohort study" was published in 2016. Journal: J Orthop Surg Res.

# Disorder-related risk factors for revision total hip arthroplasty after hip hemiarthroplasty in displaced femoral neck fracture patients: a nationwide population-based cohort study

**DOI:** 10.1186/s13018-016-0400-3

**Published:** 2016-06-08

**Authors:** Chun-Hao Tsai, Chih-Hsin Muo, Chih-Hung Hung, Tsung-Li Lin, Ta-Ii Wang, Yi-Chin Fong, Horng-Chaung Hsu

**Affiliations:** Department of Orthopedic Surgery, China Medical University Hospital, #91 Hsueh-Shih Road, Taichung, 404 Taiwan; School of Medicine, China Medical University, Taichung, Taiwan; Graduate Institute of Clinical Medicine, China Medical University, Taichung, Taiwan; Management Office for Health Data, China Medical University Hospital, Taichung, Taiwan; Tainan Municipal An-Nan Hospital-China Medical University, Tainan, Taiwan; China Medical University Beigang Hospital, Yunlin, Taiwan; School of Chinese Medicine, China Medical University, Taichung, Taiwan

## Abstract

**Background:**

The choice of primary hip hemiarthroplasty or total hip arthroplasty for displaced femoral neck fracture is still controversial. Revision hip arthroplasty not only increases risk and cost but also could result in worse outcome. Determining the risk factors for revision can help inform medical decision-making and aid in risk stratification of publicly reported outcomes. Therefore, we conducted a nationwide population-based study to identify the disease-related risk factors and construct a risk score nomogram to predict revision surgery.

**Methods:**

Records of all 68,030 femoral neck fracture patients receiving partial hemiarthroplasty (HA) in 2000–2010, with no total hip arthroplasty (THA) or revision HA history, were collected from the National Health Insurance Research Database. Cox proportional hazard regression was used to estimate the risk of revision hip replacement (RHA). The score of each risk factor was the quotient of the regression coefficient of the variable by the regression coefficient for a 10-year increase in age. The predictive accuracy was tested using the area under the receiver operating characteristic curve (AUROC).

**Results:**

The revision risk for hemiarthroplasty increased in male, those with schizophrenia and end-stage renal disease patients had 1.58-, 1.88-, and 1.74-fold revision HA risk (95 % confidence interval (CI) = 1.40–1.78, 1.26–2.79, and 1.29–2.34, respectively). In a predictive model, the cumulative risk score ranged from 0 to 13 with a 5.08 to 91.82 % 10-year predicted RHA risk. The percentage of AUROC for 10-year RHA risk in nomogram was 61.9 (95 % CI = 60.0–63.4).

**Conclusions:**

Males, schizophrenia and end-stage renal disease patients have higher risk of revision surgery after hemiarthroplasty for femoral neck fracture.

The article "Disorder-related risk factors for revision total hip arthroplasty after hip hemiarthroplasty in displaced femoral neck fracture patients: a nationwide population-based cohort study" was published in 2016. Journal: J Orthop Surg Res.

## Background

With the rapid development of the aging population, the total number of patients worldwide with hip fracture is predicted to rise to 6.26 million per year by 2050 [1]. Based on location, femoral neck fractures account for 45 to 53 % of hip fractures. The three major treatments for femoral neck fractures in clinical practice are internal fixation, hemiarthroplasty (HA), and total hip arthroplasty (THA) [2, 3]. While internal fixation applies to undisplaced intracapsular fractures [4], the other two operative methods are advisable for displaced fractures in the elderly [5]. Since HA is a standardized surgical method that allows early weight bearing and recovery, it has become an established procedure with low risk of postoperative complications. Nonetheless, higher physical demands, even in older adults, occasionally necessitate conversion surgery to THA; this processes likely to increase both the possible risks and the associated costs [6, 7]. While debate continues on whether primary THA or HA is best for displaced femoral neck fracture [6, 8–10], the high complication rate of revision HA in comparison with THA is clearly known [11].

Therefore, it has become critical to determine the specific risk factors associated with the conversion of HA to revision hip replacement (RHA), to better assess the relative risks of each surgical procedure. The few studies of the risk factors associated with conversion to THA for hemiarthroplasty have identified several risk factors, such as younger age and male gender [12]. However, the weight of each risk factor has not yet been determined. Thus, we conducted a population-based, case-control study using the nationwide population-based database of a universal insurance program to evaluate the disease-related risk factors for conversion of HA to THA in femoral neck fracture in older adults.

## Methods

### Data source

The Taiwan Bureau of National Health Insurance (TBNHI) set up a single-payer National Health Insurance (NHI) Program on March 1, 1995. Almost all residents in Taiwan join this program. TBNHI commissioned the National Health Research Institutes to maintain the National Health Insurance Research Databases (NHIRDs) derived from the NHI program. We obtained from the NHIRDs data on all inpatient claims from 1996 to 2011. To be in compliance with the Personal Information Protection Act, the insurance information was de-identified and the scientists signed an agreement that they had no intention of obtaining personal information. This study was approved by the local institutional review board. The identification of disease was based on the International Classification of Diseases, Ninth Revision, Clinical Modification (ICD-9-CM) codes in the NHIRDs.

The article "Disorder-related risk factors for revision total hip arthroplasty after hip hemiarthroplasty in displaced femoral neck fracture patients: a nationwide population-based cohort study" was published in 2016. Journal: J Orthop Surg Res.

### Study subjects and end-points

We collected adult patients with a new diagnosis of femoral neck fracture (ICD-9-CM code 820) who received partial hip arthroplasty (HA, ICD-9-operation code 81.52) in 2000–2010 (*N* = 68,755). The date of HA treatment was defined as the index date. Patients who had received total hip replacement (ICD-9-operation code 81.51, *n* = 592) or RHA (ICD-9-operation code 81.53, *n* = 133) before the index date were excluded. All study subjects were followed from the index date to the date of RHA treatment. Those without RHA treatment were followed until the date of withdrawal from the program or the end of 2011.

For the prediction model, we randomly assigned HA patients to either a derivation group or a validation group in a 3:1 ratio.

### Risk factors

The risk factors included age, gender, and comorbidity. Comorbidities assessed (using ICD-9-CM codes) included diabetes (250), osteoporosis (733.0, V17.81, V82.81), rheumatoid arthritis (RA; 714), cancer (140–208), chronic obstructive pulmonary disease (COPD; 491,492, 496), previous osteoarthritis hip (715.5), end-stage renal disease (ESRD; 585), systemic lupus erythematosus (SLE; 710.0), ankylosing spondylitis (720), obesity (278.0), extrinsic asthma (493.0), human immunodeficiency virus (HIV; 042, V08, 795.71), atherosclerosis (440), smoking (350.1 and 649.0), psoriasis (696), viral hepatitis (070), depression (296.2, 296.3, 296.82, 300.4, 311), schizophrenia (295), heart failure (428), urinary tract infection (UTI; 599.0), ischemic heart disease (410–414), dementia (290, 294.1, and 331.0–331.2), and alcoholism (291, 303, 305.00–305.03, 790.3, V11.3). All comorbidities were defined before the index date.

### Statistical analysis

#### Incidence of RHA and RHA-associated risk factors

The incidence of RHA (per 1000 person-years) was determined in patients by age, gender, and comorbidity. Cox proportional hazard regression was used to estimate the hazard ratios (HRs) and 95 % confidence interval (CI) of RHA and the RHA-associated risk factor. Multivariable modeling was used, controlling for significant factors using crude Cox proportional hazard regression.

#### Prediction model

In future analysis, the prediction model was developed according to those risk factors identified as significant in this study. The score of each risk factor was the quotient of the regression coefficient of the variable by the regression coefficient for a 10-year increase in age. The cumulative risk score was the sum of the score of each risk factor. The area under the receiver operating characteristic curve (AUROC) of the nomogram was used to test the association of factors with RHA treatment using logistic regression. In future analysis, the patients were grouped into three groups based on risk scores: low (risk score 0–2), median (risk score 3–4), and high (risk score 5+). We plotted the cumulative incidence among risk score groups by Kaplan-Meier analysis in derivation and validation cohort. All statistical analyses were performed using the SAS software package SAS (version 9.4 for windows; SAS Institute, Cary, NC).

The article "Disorder-related risk factors for revision total hip arthroplasty after hip hemiarthroplasty in displaced femoral neck fracture patients: a nationwide population-based cohort study" was published in 2016. Journal: J Orthop Surg Res.

## Results

All 68,030 femoral neck fracture patients who received hip hemiarthroplasty (HA) were selected for this study. Most patients were older than 70 years (80.8 %) and the mean age was 77.3 years (standard deviation = 9.26, Table 1). Most HA patients were female (65.0 vs. 35.0 %). The 10 most prevalent comorbidities in HA patients were diabetes (23.7 %), ischemic heart disease (18.2 %), UTI (17.9 %), COPD (10.6 %), heart failure (8.13 %), cancer (7.62 %), ankylosing spondylitis (5.42 %), osteoporosis (4.89 %), dementia (3.52 %), and ESRD (2.88 %).

**Table 1:** Incidence and hazard ratio for revision hip replacement and associated risk factor

	*n*				(%)	Event no.	PY	Rate^a^	Crude HR (95 % CI)	Adjusted HR (95 % CI)
Total	68,030					1114	238,875	4.66		
Age, year										
20–29	53				(0.08)	9	260	34.57	30.9 (13.4–71.5)***	23.6 (10.2–54.7)***
30–39	158				(0.23)	11	832	13.23	12.0 (5.43–26.4)***	8.52 (3.85–18.9)***
40–49	499				(0.73)	25	2302	10.86	9.49 (4.93–18.3)***	6.90 (3.56–13.4)***
50–59	1862				(2.74)	63	7908	7.97	6.65–3.73 (11.9)***	5.48 (3.06–9.82)***
60–69	10,492				(15.4)	257	45,526	5.65	4.77 (2.79–8.17)***	4.35 (2.54–7.46)***
70–79	26,868				(39.5)	458	101,757	4.50	3.59 (2.11–6.12)***	3.38 (1.99–5.76)***
80–89	24,095				(35.4)	277	71,159	3.89	2.80 (1.64–4.80)***	2.73 (1.60–4.68)***
≥90	4003				(5.88)	14	9132	1.53	1.00	1.00
Mean (SD)	77.3				(9.26)					
Gender										
Women	44,241				(65.0)	614	163,685	3.75	1.00	1.00
Men	23,789				(35.0)	500	75,190	6.65	1.69 (1.50–1.90)***	1.58 (1.40-1.78)***
Comorbidity										
Diabetes										
No	51,877			(76.3)		861	191,518	4.50	1.00	
Yes	16,153			(23.7)		253	47,357	5.34	1.09 (0.95–1.26)	
Osteoporosis										
No	64,702			(95.1)		1057	228,211	4.63	1.00	
Yes	3328			(4.89)		57	10,664	5.35	1.11 (0.85–1.45)	
RA										
No	67,472			(99.2)		1099	236,796	4.64	1.00	
Yes	558			(0.82)		15	2079	7.21	1.57 (0.94–2.61)	
Cancer										
No	62,848			(92.4)		1038	226,145	4.59	1.00	
Yes	5182			(7.62)		76	12,730	5.97	1.14 (0.90–1.44)	
COPD										
No	60,853			(89.4)		1008	219,410	4.59	1.00	
Yes	7177			(10.6)		106	19,465	5.45	1.07 (0.88–1.31)	
ESRD										
No	66,073		(97.1)			1068	234,698	4.55	1.00	1.00
Yes	1957		(2.88)			46	4177	11.01	1.99 (1.48–2.68)***	1.74 (1.29–2.34)***
SLE										
No	67,963		(99.9)			1112	238,679	4.66	1.00	
Yes	67		(0.10)			2	196	10.19	2.03 (0.51–8.14)	
Ankylosing spondylitis										
No	64,346		(94.6)			1059	228,091	4.64	1.00	
Yes	3684		(5.42)			55	10,785	5.10	1.02 (0.78–1.34)	
Extrinsic asthma										
No	67,850		(99.7)			1112	238,299	4.67	1.00	
Yes	180		(0.26)			2	576	3.47	0.72 (0.18–2.89)	
HIV										
No	68,022		(99.9)			1114	238,853	4.66	1.00	
Yes	8		(0.01)			0	22	0.00	––	
Atherosclerosis										
No	67,550		(99.3)			1106	237,521	4.66	1.00	
Yes	480		(0.71)			8	1355	5.91	1.17 (0.58–2.35)	
Psoriasis										
No	67,898		(99.8)			1112	238,505	4.66	1.00	
Yes	132		(0.19)			2	370	5.40	1.09 (0.27–4.36)	
Viral hepatitis										
No	66,212		(97.3)			1080	234,523	4.61	1.00	1.00
Yes	1818		(2.67)			34	4353	7.81	1.46 (1.04–2.06)*	1.30 (0.92–1.83)
Depression										
No	66,091	(97.2)				1081	232,874	4.64	1.00	
Yes	1939	(2.85)				33	6002	5.50	1.12 (0.79–1.59)	
Schizophrenia										
No	67,399	(99.1)				1088	236,468	4.60	1.00	1.00
Yes	631	(0.93)				26	2408	10.80	2.43 (1.65–3.58)***	1.88 (1.26–2.79)**
Heart failure										
No	62,500	(91.9)				1035	22,478	4.59	1.00	
Yes	5530	(8.13)				79	13,397	5.90	1.11 (0.89–1.40)	
UTI										
No	55,877	(82.1)				936	204,007	4.59	1.00	
Yes	12,153	(17.9)				178	34,869	5.10	1.2 (0.87–1.19)	
Ischemic heart disease										
No	55,681	(81.9)				915	203,038	4.51	1.00	
Yes	12,349	(81.9)				199	35,837	5.55	1.13 (0.97–1.32)	
Dementia										
No	65,633	(96.5)				1091	231,906	4.70	1.00	1.00
Yes	2397	(3.52)				23	6969	3.30	0.65 (0.43–0.98)*	0.71 (0.47–1.07)

*PY* person-years, *HR* hazard ratio, *CI* confidence interval, *SD* standard deviation, *RA* rheumatoid arthritis, *COPD* chronic obstructive pulmonary disease, *ESRD* end-stage renal disease, *SLE* systemic lupus erythematosus, *HIV* human immunodeficiency virus, *UTI* urinary tract infection

*p < 0.05; **p < 0.01; ***p < 0.001

^a^Per 1000 person-years

After a cumulative 12-years follow-up, 1114 patients received RHA treatment, with an incidence of 4.66 per 1000 person-years (Table 1). In multivariable Cox proportional hazard regression, the RHA risk decreased with aging from 23.6 to 2.73 in those aged 20-29 to 80-89 years, respectively, compared with those aged ≥90 years (95 % CI = 10.2-54.7 and 1.60-4.68, respectively). Compared with women, men had a significantly higher RHA risk (HR = 1.58, 95 % CI = 1.40–1.78). RHA-associated risk factors for the total cohort were schizophrenia (HR = 1.88, 95 % CI = 1.26–2.79) and ESRD (HR = 1.74, 95 % CI = 1.29–2.34).

The article "Disorder-related risk factors for revision total hip arthroplasty after hip hemiarthroplasty in displaced femoral neck fracture patients: a nationwide population-based cohort study" was published in 2016. Journal: J Orthop Surg Res.

Table 2 presents the distribution between derivation (75.0 %) and validation (25.0 %) cohort. There was no significant difference of age, gender, ESRD and schizophrenia between two groups. In derivation cohort, the risk score decreased one point with every 10 years of age increasing; for example, the risk score was 7 for patients aged 20–29 years, 6 for those 30–39 years, 5 for those 40–49 years, and so on (Table 3). The risk score was 2 for men, those with ESRD and schizophrenia patients. The percentage of AUROC for 10-year RHA risk in nomogram was 61.9 (95 % CI = 60.0–63.4). In the prediction model, the cumulative risk score ranged from 0 to 13 with a 5.08 to 91.82 %10-year predicted RHA risk (Fig. 1).

**Table 2:** Distribution of predictor between derivation and validation cohort

	Derivation cohort		Validation cohort		
	*N* = 51021 (75.0 %)		*N* = 17009 (25.0 %)		
	*n*	%	*n*	%	Chi-square *p* value
Age, year					0.98
20–29	40	0.08	13	0.08	
30–39	113	0.22	45	0.26	
40–49	371	0.73	128	0.75	
50–59	1388	2.72	474	2.79	
60–69	7878	15.4	2614	15.4	
70–79	20,177	39.6	6691	39.3	
80–89	18,047	35.4	6048	35.6	
≥ 90	3007	5.89	996	5.86	
Gender					0.97
Women	33,182	65.0	11,059	65.0	
Men	17,839	35.0	5959	35.0	
Comorbidity					
ESRD	1493	2.93	464	2.73	0.18
Schizophrenia	455	0.89	176	1.03	0.09

*ESRD* end-stage renal disease

**Table 3:** Incidence and hazard ratio for revision hip replacement and associated risk factor in derivation cohort

	HR (95 % CI)	Regression coefficient	*p*	Risk score
Age, year				
20–29	40.4 (16.0–10.2)	3.700	< 0.0001	7
30–39	12.3 (4.85–31.0)	2.506	< 0.0001	6
40–49	8.40 (3.76–18.8)	2.128	< 0.0001	5
50–59	6.44 (3.14–12.2)	1.862	< 0.0001	4
60–69	4.92 (2.52–9.62)	1.593	< 0.0001	3
70–79	3.97 (2.05–7.71)	1.380	< 0.0001	2
80–89	3.38 (1.74–6.59)	1.218	0.0003	1
≥ 90	Ref.	0		0
Gender				
Women	Ref.	0		0
Men	1.57 (1.36–1.80)	0.449	< 0.0001	2
ESRD				
No	Ref.	0		0
Yes	1.72 (1.22–2.43)	0.542	0.002	2
Schizophrenia				
No	Ref.	0		0
Yes	1.84 (1.15–2.96)	0.611	0.01	2
Baseline disease–free probability				
At 10 years	96.89			
AUROC % (95 % CI)	61.9 (60.0–63.4)			

*HR* hazard ratio, *CI* confidence interval, *AUROC* the area under the receiver operating characteristic curve

**Fig. 1:** Nomograms for the prediction of the RHA risk

Figure 2 presents cumulative incidence of RHA in different risk score groups. In derivation cohort, the cumulative incidences of RHA were 2.03, 3.85, and 6.06 % in low, median, and high after 10 years follow-up, respectively. In validation cohort, patients with higher risk score had highest cumulative incidence of RHA (6.24 %) and followed by median and low group (3.86 and 1.85 %).

**Fig. 2:** Cumulative incidence for revision hip replacement among different risk score groups: low (risk score 0–2), median (risk score 3–4), and high (risk score 5+) in derivation (**a**) and validation (**b**) cohort

The article "Disorder-related risk factors for revision total hip arthroplasty after hip hemiarthroplasty in displaced femoral neck fracture patients: a nationwide population-based cohort study" was published in 2016. Journal: J Orthop Surg Res.

## Discussion

The current study revealed that the rate of RHA for primary HA for femoral neck fracture is 4.67 per 1000 person-years. Several risk factors, such as age, gender, ESRD, and schizophrenia, were identified. We also assessed the contribution of each factor to help clinicians predict future revision rate.

Traditionally, surgeons have preferred HA over THA because of concerns about the increased risk of complications of the more complex THA. However, more current data has showed no significant differences in the complication rates of patients undergoing HA versus THA [2, 9, 13, 14]. Moreover, the literature shows a lower risk of reoperation after THA compared with HA [6, 12, 14–16] and better functional outcomes for patients after THA versus HA [6, 8–10, 13, 14, 16, 17].

HA comes with considerable risk of reoperation with conversion to THA [18, 19]. Finite element mode study has proven that HA increases the biomechanical stresses on the acetabular bone that would result in migration of the head and destruction of the acetabulum [20]. Several studies found significant acetabular wear in up to 67 % of cases [21, 22], quantified at an average rate of 0.7 mm per year [22]. The inability to restore the femoral offset is also a factor [23], impairing the ability to balance tissue tension. However, THA is not suitable for every patient, including those with multiple morbidities or those with limited life expectancy [24]. The disadvantages of THA include greater blood loss and higher costs compared with HA [13]. Despite higher initial costs, the overall costs of THA are lower.

Young age and male gender are well-identified risk factors for revision HA surgery [12], but no literature has described schizophrenia or ESRD as risk factors for revision HA surgery. Schizophrenia has been associated with higher odds of perioperative blood transfusion, adverse events, and non-routine discharge following total joint arthroplasty (TJA) [25, 26] or spine surgery [27]. ESRD is also a risk factor for perioperative allogeneic blood transfusions [28], as it increased both mortality and the complication rate in TJR [29, 30].

Risk equations and risk functions have been widely applied for patient counseling, clinical diagnosis, risk stratification, treatment selection, and prognosis prediction; these have especially been useful in medical fields such as cardiovascular disease [31], hepatic disease [32, 33], and cancer [34, 35]. Most risk score systems used in orthopedic surgery are constructed according to the preoperative damage condition [36, 37], bony destruction [38], or postoperative fixation status [39]. In preoperative assessment of displaced femoral neck fracture without complicated bony destruction, using demographic data and underlying comorbidity is an easy way to predict risk of revision. The nomogram of this study does not require complex calculations but allows surgeons to estimate the impact of demographic risk factors by easily adding the risk score. It helps facilitate clinician communication with patients about risk prediction and decision-making.

The article "Disorder-related risk factors for revision total hip arthroplasty after hip hemiarthroplasty in displaced femoral neck fracture patients: a nationwide population-based cohort study" was published in 2016. Journal: J Orthop Surg Res.

Our study has several limitations. First, we relied on NHIRDs to identify revisions and risk factors for revision HA surgery. Because the ICD-9 coding is representative of diseases, but not of the life style neither the physical finding. We are not able to analyze the population of smoker, alcohol use, and obesity because the insurance system only could code when the patients ask for medical treatment, which means the life style has threaten the health. Therefore, our data cannot show the risk of RHA in smoker, alcohol use, either BMI for obesity. However, smoke is a risk factor to infection [40], early failure, and revision surgery in total hip arthroplasty. Dislocation risk will be increased in alcoholism after total hip arthroplasty [41].

Second, the most common cause of revision hip replacement is loosening of the prosthesis (Table 4); however, there is no coding about primary surgery method or revision method. Therefore, we were not able to assess the surgical approach and type of prosthesis used (including retained stem, cemented, or noncemented prosthesis). Surgical approach would play a role in dislocation rate after hemiarthroplasty. Direct anterior [42, 43] or anteriorlateral approach has less dislocation rate that posterior approach [44, 45]. Both cemented and uncemented stem have good functional results in hip hemiarthroplasty for displaced femoral neck fractures [46]. But the uncemented hemiarthroplasty has high risk of postoperative periprosthetic femoral fractures to reoperation [47–50]. However, previous investigators have reported a reasonable correlation between administrative claims and the clinical record when evaluating causes and types of revision TJA procedures [13]. Third, our study was a retrospective cohort study rather than a prospective randomized trial. Besides, the life style pattern and physical characters of people vary in different countries. The medical insurance data result may be not as the same as other country due to different socioeconomic situations between nations. There may be some risk factors not significant in one population but may play an important role in others due to risk exposure cases number, especially in life style. Our result would not be representative of other country or population. However, the use of a population-based data set allows for the enrollment of a large number of patients and is highly representative of the risk factors of diseases found in a general population. This study reveals the importance of associated diseases affect the outcome in hip hemiarthroplasty for femoral neck fracture. In the future, we still need more cases form other population for comparison and meta-analysis to find out more risk factor or related disease.

The article "Disorder-related risk factors for revision total hip arthroplasty after hip hemiarthroplasty in displaced femoral neck fracture patients: a nationwide population-based cohort study" was published in 2016. Journal: J Orthop Surg Res.

**Table 4:** Top ten reasons due to revision hip replacement (*N* = 1114)

Disease (ICD-9-CM)	Percentage
Mechanical complication of internal orthopedic device, implant, and graft (996.4)	62.6
Infection and inflammatory reaction due to internal prosthetic device, implant, and graft (996.6)	8.71
Other complications of internal (biological) (synthetic) prosthetic device, implant, and graft (996.7)	3.50
Shaft or unspecified part, closed (821.0)	2.69
Acquired deformities of hip (736.3)	2.60
Peritrochanteric fracture, closed (820.2)	2.60
Unspecified part of neck of femur, closed (820.8)	2.42
Osteoarthrosis, localized, not specified whether primary or secondary (715.3)	1.97
Pyogenic arthritis (711.0)	1.53
Mechanical complication of other specified prosthetic device, implant, and graft (996.5)	1.44

Finally, our results are limited to risk factors for failures that occur within the 10 years after primary HA, and therefore, it is unclear whether the same or other risk factors are associated with longer term follow-up. However, the impact of patient comorbidities on the risk of revision after HA has important clinical and policy implications for the health care system. Finally, these HAs were for femoral neck fracture only; our study does not address the risk factors for HA for osteonecrosis of the femoral head.

## Conclusions

In conclusion, to assess the future risk of revision, a risk score system was developed, based on patient demographics and comorbidities. Although the permissible degree of postoperative activity depends entirely on the general health status of each patient, the current result scan help with arranging earlier rehabilitation and developing an appropriate follow-up program to prevent early complications.

## Abbreviations

AUROC, area under the receiver operating characteristic curve; CI, confidence interval; HA, hemiarthroplasty; ICD-9-CM, International Classification of Diseases, Ninth Revision, Clinical Modification; NHI, National Health Insurance; RHA, revision hip arthroplasty; THA, total hip arthroplasty
